The article "Lentivirus-Mediated siRNA Targeting ER-α Inhibits Tumorigenesis and Induces Apoptosis in Hepatocarcinoma Cells" was retracted in 2020. Reasons: errors in the analysis; plagiarized text; duplicated images; overlap with other authors' work.

# Lentivirus-Mediated siRNA Targeting ER-*α* Inhibits Tumorigenesis and Induces Apoptosis in Hepatocarcinoma Cells

**DOI:** 10.1155/2015/490681

**Published:** 2015-08-27

**Authors:** Ping Jiang, Jun Cao, Wen-Hui Bai

**Affiliations:** Department of General Surgery, Zhongnan Hospital of Wuhan University, 169 Donghu Road, Wuhan, Hubei 430071, China

## Abstract

*Background and Objectives*. Estrogen receptor-*α* (ER-*α*) plays important roles in hepatocarcinogenesis. Recent studies have shown that ER-*α* could lead to cell cycle progression or inhibition of apoptosis. To better understand the role of ER-*α*, RNA interference (RNAi) was used to inhibit ER-*α* expression in the human hepatocellular carcinoma (HCC) cells. *Methods*. Lentivirus-mediated ER-*α* small interfering RNA (siRNA) was transfected into HCC cells Hep3B. ER-*α* expression was monitored by real-time polymerase chain reaction (PCR) and western blot. Cell proliferation, apoptosis, and invasion were examined by methyl thiazol tetrazolium (MTT), flow cytometry (FCM), and invasion assay, respectively. *Results*. ER-*α* siRNA efficiently downregulated the expression of ER-*α* in Hep3B cells at both mRNA and protein levels in a time-dependent manner. ER-*α* siRNA also inhibited cell proliferation and reduced cell invasion (compared with other groups, *P* < 0.05, resp.). Furthermore, knockdown of ER-*α* slowed down the cell population at S phase and increased the rate of apoptosis (*P* < 0.05, resp.). *Conclusion*. ER-*α* knockdown suppressed the growth of HCC cells. Thus, ER-*α* may play a very important role in carcinogenesis of HCC and its knockdown may offer a new potential gene therapy approach for human liver cancer in the future.

## 1. Introduction

Hepatocellular carcinoma (HCC) is one of the most common malignant tumors that seriously threaten the human health. Its poor prognosis makes it the third leading cause of cancer-related mortality and its incidence has a rising trend [1]. Epidemiological reports indicate that, regardless of etiologies, the incidence of HCC is higher in males than in females [2]. Clinical observations also reveal that chronic liver disease progresses more rapidly to cirrhosis in males than females and therefore cirrhosis that leads to HCC development is largely considered to be the disease of men and postmenopausal women [3]. Though this sexual dimorphism in liver cancer may be partly attributed to differences in lifestyle [4], estrogen plays an important role in HCC. However, the precise effect of estrogen in HCC remains still poorly understood and controversial. Both carcinogenic and protective effects of estrogen in the liver have been reported [3, 5, 6]. The effects of estrogens are mediated by estrogen receptors (ERs). There are two known ERs: ER-*α* and ER-*β*. The majority of the effects of estrogen are mediated by ER-*α* in the liver [7]. Abnormal ER-*α* expressions in the liver have been implicated in hepatocyte injury and may act as liver disease inducers [8]. Moreover, ER-*α* plays a role in promoting liver tumors in males. A greater extent of ER-*α* expression is found in male patients of HCC than in females [9]. Furthermore, ER-*α* was found to participate in the pathogenesis of persistent hepatitis B virus (HBV) infection which is a major risk factor of HCC [10]. We postulate that ER-*α* in liver cancer cells may act as a pivotal factor in tumorigenesis. However, there are few reports on direct detection of ER-*α* using specific knockdown method in HCC. In the present study, we describe the effective targeting of ER-*α* with siRNA in HCC cells. The siRNA were delivered using lentivirus, leading to potent knockdown of ER-*α*. We aimed to investigate the effects of ER-*α* knockdown on cell proliferation, cell cycle progression, invasion, and apoptosis in HCC cell lines.

## 2. Materials and Methods

### 2.1. Lentiviral Vectors Encoding Small Interfering RNAs Targeting ER-*α*

Three predesigned small interfering RNA (siRNA) sequences targeting the ER-*α* (GenBank accession number NM_005702) were designed by Genechem Co., Ltd., Shanghai, China. The specificity for ER-*α* disruption was determined by transfecting the three siRNAs into Hep3B and HCCLM3 cell lines using FUGENE HD according to the manufacturer's instructions (Invitrogen, Carlsbad, CA, USA). After screening to validated potential siRNAs, the ER-*α* siRNA target sequence (5′-GCCTTACAATGTACA GCAGAA-3′) was selected for the construction with lentiviral vector. A nonsilencing sequence (5′-TTCTCCGAACGTGTCACGT-3′) was used as a negative control. Construction of lentiviral vectors and vector packaging were carried out as previously described [11].

### 2.2. Cell Culture and Lentivirus Infection

This experiment was conducted in accordance with the guidelines of the Ethics Committee of Wuhan University. The Hep3B and HCCLM3 cell lines were obtained from American type culture collection (ATCC, Manassas, VA). Cells maintained in DMEM (Hyclone) and supplemented with 10% fetal bovine serum (Hyclone) at 37°C in a humidified 5% CO_2_/95% air atmosphere. Cells were then seeded in 6-well plates (at a density of 5 × 10^5^ cells/well). Lentiviral vectors were transfected into cells with LV or without siRNA sequences including ER-*α* siRNA and nonsilencing siRNA (NS siRNA) at an MOI (multiplicity of infection) of 10 when the cells reached 70% confluency. After 24 h of infection at 37°C, the medium was replaced by fresh DMEM. The cells were harvested at indicated time points.

### 2.3. Real-Time RT-PCR

Total RNA was isolated from cells by using Trizol Reagent (Invitrogen, Carlsbad, CA, USA). The synthesis of cDNA was performed by using Reverse Transcription Reagents (Promega, Madison, Wisconsin, USA). Real-time PCR was performed using SYBR GREEN I Mix (ABI, Foster City, CA, USA) and an ABI Prism 7700 sequence detection system (ABI, Foster City, CA, USA) was done according to the manufacturer's instructions. Primer sequences for ER-*α* are 5′-TGTGCAATGACTATGCTTCA-3′ (sense) and 5′-GCTCTTCCTCCTGTTTTTA-3′ (antisense). Each PCR consisted of 30 cycles (30 s at 94°C, 30 s at 60°C, and 30 s at 72°C). Differences in expression were normalized to the *β*-actin signal.

### 2.4. Western Blot Analysis

Cells from each group were collected after 24, 48, or 72 hours of incubation. Cells were lysed after infection with sodium dodecyl sulfate (SDS) sample buffer. Total protein concentration was measured using the BCA protein assay kit (Pierce, Rockford, IL) with bovine serum albumin as the standard protein. Equal amounts of protein were loaded for each lane. Samples were heated at 100°C for 5 to 10 min before loading and separated on precasted 10% SDS-polyacrylamide gels (Bio-Rad, Hercules, CA). Proteins were electrotransferred to a nitrocellulose membrane (Bio-Rad) in transfer buffer containing 48 mmol/L Tris-HCl, 39 mmol/L glycine, 0.037% SDS, and 20% methanol at 4°C for 1 h. Nonspecific binding to the membrane was blocked for 1 h at room temperature with 5% nonfat milk in TBS buffer. The membranes were incubated for 16 h at 4°C with various primary antibodies in TBS buffer containing 5% milk at the dilutions specified by the manufacturer. Antibodies were purchased from Maixin Biotech Co. (Fujian, China). Binding of primary antibodies was followed by incubation for 1 h at room temperature with the secondary horseradish peroxidase-conjugated IgG in 1% nonfat milk. *β*-actin was used as a control for equal protein loading. Positive band was analyzed by gel photodensitometry analysis software Gel pro 4.0 (Media Cybernetics, Rockville, MD).

### 2.5. Cell Viability, Proliferation, and Colony Formation Assay

Cell viability was assessed by methyl thiazol tetrazolium (MTT) assay. Cells were plated in 96-well plates containing 10% FBS. After infection with ER-*α* siRNA, NS siRNA, or LV for 0, 24, 48, or 72 hours, cells from each group were collected and plated in 96-well plates at a density of 1.0 × 10^4^ cells/well for MTT assay. Untreated cells served as control. The absorbance was measured at 570 nm. Each assay was performed in triplicate. Cell growth (mean absorbance ± standard deviation) was plotted versus time. A cell proliferation assay was done by counting cell number. Cells were plated at a density of 5.0 × 10^4^ cells/mL in 24-well plates and infected with lentivirus vectors. Cells were harvested daily and counted. As previously described [12], a soft agar colony formation assay was used to assess the growth ability of HCC cells* in vitro*. Cells were infected with lentiviral vectors encoding siRNA sequences for 24 hours. Cells were then plated on a 0.6% agarose base in six-well plates in 1 mL of DMEM medium containing 10% FBS and 0.3% agarose. Colonies > 50 *μ*m were counted 14 days after plating.

### 2.6. Flow Cytometry Analysis of Cell Cycle and Apoptosis

The effect of ER-*α* silencing on cell cycle distribution was determined by a flow cytometry analysis of the DNA content of the nuclei of the cells after staining with PI. After infection with ER-*α* siRNA, NS siRNA, or LV for 0, 24, 48, or 72 hours, Hep3B cells were washed with PBS and fixed in 70% ice cold ethanol at 4°C for at least 1 h. Untreated cells served as control. The cells were resuspended in phosphate-buffered saline (PBS) containing 100 *μ*L propidium iodide (PI) (BD Biosciences, San Jose, CA, USA) and 100 *μ*L RNase A for 30 min at 37°C, and DNA quantities in different cell cycles (G0/G1, S, and G2/M phases) were analyzed by flow cytometry (BD Biosciences).

Flow cytometry was also used to determine the apoptotic rate. Surface exposure of phosphatidylserine in apoptotic cells was quantitatively detected using the Annexin V-APC Apoptosis Detection Kit as described by the manufacturer's instruction. Briefly, after infection with ER-*α* siRNA, NS siRNA, or LV for 0, 24, 48, or 72 hours, Hep3B cells incubated with 5 *μ*L Annexin V-FITC/PI (BD Biosciences, San Jose, CA, USA) and 5 *μ*L PI for 15 min. Annexin V-positive and PI-negative cells were identified as apoptotic cells. The apoptotic rate was determined using CellQuest software (FCM, BD Biosciences, San Jose, CA, USA).

### 2.7. Cell Invasion Assay

The infected cells by ER-*α* siRNA, NS siRNA, or LV were cultured for 0, 24, 48, or 72 hours followed by treatment with 2.5% trypsin and suspended in serum-free DMEM medium at a concentration of 5 × 10^4^/mL. Cells were seeded into the upper chamber and grown in 600 *μ*L DMEM medium containing 10% FCS loaded in the lower chamber. Then the transwell chambers (Corning Costar, NY, USA) were incubated in a 37°C, 5% CO_2_/95% air, humidified incubator for 24 h. The cells on the inner surface of the filter membrane were removed. Cells on the lower surface of the membrane were stained with crystal violet and counted in five random fields by 200x magnification light microscope (Olympus, Beijing, China). Percentage of invaded cells in each group was calculated.

### 2.8. Statistical Analysis

Data are expressed as mean ± SD and processed by the statistical analysis software SPSS version 16.0 (SPSS Inc., Chicago, IL, USA). Comparisons among all groups were performed with the one-way analysis of variance (ANOVA) test or unpaired Student's *t*-test. All *P* values were two-tailed and a *P* value of less than 0.05 was considered significant. The results shown in each of the figures in this paper are representative of at least three independent experiments.

## 3. Results

### 3.1. Lentivirus-Mediated siRNA Efficiently Downregulates ER-*α* Expression in Hep3B Cells

To determine the efficiency of lentivirus-mediated siRNA for ER-*α*, real-time RT-PCR analysis was performed. As shown in Figure 1(a), expression of ER-*α* was reduced as early as 24 hours after infection of ER-*α* siRNA. Seventy-two hours after infection the relative level of ER-*α* mRNA expression in cells of ER-*α* siRNA group was significantly decreased compared with that in the other groups (*P* < 0.05, resp.). In addition, the expression of ER-*α* protein was analyzed by western blot. The amount of ER-*α* protein in cells of ER-*α* siRNA group also decreased greatly after infection of 24, 48, and 72 hours (*P* < 0.05) (Figure 1(b)). These results indicated that the lentivirus-mediated ER-*α* siRNA could efficiently downregulate ER-*α* expression in Hep3B and HCCLM3 cells.

### 3.2. Effects of ER-*α* Knockdown on Cell Proliferation

To determine whether ER-*α* knockdown by RNAi had an inhibitory effect on Hep3B and HCCLM3 cells viability, we carried out MTT assay. We found that treatment of both Hep3B and HCCLM3 cells with ER-*α* siRNA was associated with a time-dependent inhibition of cell growth, whereas no significant inhibitory effect was observed in cells treated with NS siRNA, LV, or untreated cells (Figure 2(a)). Cell proliferation was significantly inhibited at 3 days of infection (*P* < 0.01) and the average proliferation inhibition rates were 25~38% (Figure 2(b)). In addition, treatments with ER-*α* siRNA inhibit Hep3B and HCCLM3 cell colony formation in soft agar by 50~60% (Figure 2(c)). These data suggest that ER-*α* played a critical role in hepatocarcinoma cell proliferation.

### 3.3. Effects of ER-*α* Knockdown on Cell Cycle and Apoptosis

In order to find out whether ER-*α* siRNA delays cell proliferation partly through regulation of cell cycle, we then examined cell cycle distribution by flow cytometry. Compared with cells in the other groups, cells infected with ER-*α* siRNA group showed a substantial decrease in S-phase (*P* < 0.05, resp.) (Figure 3(a)). We also carried out an Annexin V Apoptosis Assay to determine the apoptotic effect of ER-*α* siRNA on Hep3B and HCCLM3 cells. In time course experiment, silencing of ER-*α* significantly increased the percentage of apoptotic cells compared with the other groups (*P* < 0.05, resp.) (Figure 3(b)). Compared with the control group and LV group, NS siRNA did not significantly increase cell apoptosis (*P* > 0.05, resp.).

These results indicated that ER-*α* knockdown inhibited HCC cell proliferation by inducing cell cycle arrest and apoptosis.

### 3.4. Effect of ER-*α* Knockdown on Cell Invasion

We investigated the effects of ER-*α* knockdown on invasion of Hep3B and HCCLM3 cells. In Hep3B cells, we found that ER-*α* siRNA infected cells showed a significant decreased invasion compared with cells in untreated group (50 ± 17 versus 201 ± 36, *P* = 0.021), LV group (50 ± 17, versus 214 ± 45, *P* = 0.016), and NS siRNA group (50 ± 17 versus 210 ± 34, *P* = 0.018) (Figure 4). NS siRNA group showed no significant differences in cell invasion compared with the control group (210 ± 34 versus 201 ± 36, *P* = 0.22) and LV group (210 ± 34 versus 214 ± 45, *P* = 0.034). Similar findings have been observed in HCCLM3 cells. The number of invaded cells was significantly decreased in ER-*α* siRNA infected cells compared to other groups (*P* < 0.05, resp.).

## 4. Discussion

In our study, lentivirus-mediated RNAi was used to silence ER-*α* in the human HCC cell lines Hep3B. The siRNA targeting ER-*α*, expressed from the recombinant lentivirus, induced efficient inhibition of endogenous ER-*α* mRNA and protein expression in the cell line. Simultaneously, inhibition of ER-*α* expression led to decreased proliferation, invasion capacity, and apoptosis of these tumor cells. Thus, this study is to observe and confirm a crucial role of ER-*α* in the progression of HCC, showing that ER-*α* may act as an important role in promoting HCC.

The role of ERs in liver diseases has become evident for recent decades. There are two isoforms of ERs, ER-*α* and ER-*β*. Some studies have found that liver ER-*α* levels increase when HCC develops [13]. Estrogen-bound ER-*α* could lead to cell cycle progression and inhibition of apoptosis [14]. Results from a mouse model of HCC also indicate that ER-*α* plays a role in the promotion of liver tumors in males [15]. However, in sharp contrast, recent studies demonstrated that estrogen was able to repress HCC growth and metastasis [16, 17]. Studies of chemical carcinogenesis also suggested that ER-*α* might modulate HCC risk by inhibiting the malignant transformation of preneoplastic liver cells. These contradictory results strongly suggest that ER-*α* mutated in HCC cells. Likely, in breast cancer (classical estrogen-dependent tumor), the progression from hormone dependence to hormone independence and the contemporary development of a more aggressive phenotype have been associated with the onset of variant ER-*α* (vER) [18]. Previous studies showed that normal liver expresses almost exclusively normal wild type ER (wtER) while, in HCC, vER can be the only expressed form [13, 19, 20]. In HCC cells, the abnormal vER lost function during disease progression and has been implicated in stimulating hepatocyte injury [8]. High rate of vER-*α* was found to correlate with a higher clinical aggressiveness of the tumor in comparison with the tumors characterized by wtER-*α* transcript [21]. The presence of vERs is able to influence the natural history of patients with HCC by regulating tumor growth as well as patient survival [22]. Megestrol, a potent antagonist of both vER and wtER, was able to influence favorably the course of HCC, which is consistent with results of our present study. However, the underlying mechanism of vER-*α* in HCC progression remains unclear. Miceli et al. demonstrated that HCC cells expressed high level of vER but no wtER; the vER in HCC may upregulate amphiregulin expression and increase malignant cell proliferation [22]. Han et al. found that, in hepatoma cells, vER was shown to interfere with the transcriptional activity of normal wtER [23]. In our further study, we are going to determine the phenotypes of ER-*α* and the underlying molecular pathways of ER-*α* in HCC cells.

In our research, siRNA is used to silence the target gene (ER-*α*). It has become a new method for the study of gene function as well as for the gene therapy [24]. At present, the most common method used in laboratory was liposome infection, which delivered siRNA to cells and then the corresponding function was played. However, studies showed that liposomes and other carriers had a great toxicity to cells and the infection efficiency was low and not long-lasting [25]. To overcome poor infection efficiency and other defects, we used the lentiviral vector as a delivery tool for siRNAs to silence genes, which had advantages in the large capacity of transfer gene fragment, a long time expression of target gene and little immune response. Our results showed that the rate of lentivirus-mediated siRNA infection reached 80% which is much higher than that of liposome transfection we once used in our pretest. In previous studies, other target genes such as Med19 [26], RHBDD1 [27], and Wtp53-pPRIME-miR30 [28] were also specifically and effectively silenced by lentivirus-mediated siRNA, leading to significant antitumorigenesis effects* in vivo* or even* in vitro*. These results suggest that lentivirus-mediated siRNA system has good targeting ability and may serve as a potent therapeutic method for liver cancer.

## 5. Conclusion

It is demonstrated for the first time that ER-*α* silencing by lentivirus-mediated siRNA inhibits Hep3B and HCCLM3 cell proliferation via inducing cell cycle arrest and cell apoptosis and also reduces invasion and proliferation of HCC cells. Therefore, we can suppose that ER-*α* plays role in HCC tumorigenesis and is a potent molecular target for liver cancer therapy.

## Figures and Tables

**Figure 1:** Effects of siRNA on ER-*α* expression in Hep3B and HCCLM3 cells. ER-*α* expression levels were analyzed by (a) real-time PCR and (b) western blot at the different times after virus infection. LV: lentivirus; NS siRNA (NS): nonsilencing siRNA; cells untreated served as control. Data were expressed as mean ± SD. Compared with other groups, ^#^ *P* < 0.05, ^##^ *P* < 0.01; compared with other time points, ^*∗*^ *P* < 0.05, ^*∗∗*^ *P* < 0.01.

**Figure 2:** Effect of ER-*α* knockdown on cell proliferation. Hep3B and HCCLM3 cells were infected with ER-*α* siRNA, nonsilencing siRNA (NS siRNA), or lentivirus (LV). Cells untreated served as control. After 0, 24, 48, or 72 hours of incubation, cell viability was performed by MTT assay (a); a cell proliferation assay was done by counting cell number at 1, 3, 5, and 7 days after infection (b); a soft agar colony formation assay was carried out 14 days after infection to assess the growth ability of cells (c). Compared with other groups, ^#^ *P* < 0.05, ^##^ *P* < 0.01.

**Figure 3:** Effects of ER-*α* knockdown on cell cycle and apoptosis. (a) Cell cycle pattern was analyzed 24, 48, and 72 hours after the infection by a flow cytometry with MODFIT software data interpretation. ER-*α* knockdown caused significant decrease in distribution of S phase in both Hep3B and HCCLM3 cell lines. (b) Hep3B cells and HCCLM3 treated with ER-*α* siRNA, NS siRNA, or LV and untreated cells were incubated for 24, 48, and 72 hours, respectively. Cells untreated served as control. Compared with other groups, ^#^ *P* < 0.05, ^##^ *P* < 0.01.

**Figure 4:** The effects of ER-*α* knockdown on cell invasion. The invasive ability was significantly weakened in Hep3B and HCCLM3 cells treated with ER-*α* siRNA compared with other groups; cells untreated served as control.
